The article "Acute pancreatitis associated with the antibiotic levofloxacin: A rare case report" was retracted in 2026. Reasons: plagiarism; overlap with other authors' work.

# Acute pancreatitis associated with the antibiotic levofloxacin: A rare case report

**DOI:** 10.1002/ccr3.8186

**Published:** 2023-11-27

**Authors:** Pugazhendi Inban, Virali Gulla, Aarfa Devani, Chinaza Mercy Akuma, Chengala Ananyaa Gowthavaram, Akbar Hussain, Lynn Lat Lat Aung, Neel Jadav, Bansi Savaliya, Taha Sajjad, Aadil Mahmood Khan, Ogbonnaya Akuma, Anasonye Emmanuel Kelechi

**Affiliations:** ^1^ Department of General Medicine Government Medical College, Omandurar Chennai India; ^2^ Internal Medicine Sri Padmavathi Medical College, SVIMS Tirupati India; ^3^ Department of Internal Medicine Malla Reddy Institute of Medical Sciences Hyderabad India; ^4^ Chamberlain University College of Health Professions Chicago Illinois USA; ^5^ Internal Medicine Malla Reddy Institute of Medical Sciences Hyderabad Telangana India; ^6^ Internal Medicine Jinnah Sindh Medical University Karachi City Sindh Pakistan; ^7^ College of Medicine MAHSA university Kaulalampur Malaysia; ^8^ Internal Medicine Pramukh Swami Medical College Valsad India; ^9^ Crimean Federal University Simferopol Russia; ^10^ Medical Education Mount Vista Medical Centre PHOENIX Arizona USA; ^11^ Department of Cardiology University of Illinois Chicago Illinois USA; ^12^ Ebonyi State University Abakaliki Nigeria; ^13^ Texila American University Georgetown Guyana

**Keywords:** abdominal ultrasonography, computed tomography, drug‐induced acute pancreatitis, fluoroquinolone, levofloxacin, photosensitivity

## Abstract

Drug‐induced acute pancreatitis is a potentially ignored diagnosis that must be precisely valued. Drug‐induced acute pancreatitis can be considered the third common cause of acute pancreatitis after ruling out alcohol and gallstones. Levofloxacin belongs to a class of fluoroquinolone antibiotics used for treating various infections. Besides photosensitivity and liver toxicity, levofloxacin can induce acute pancreatitis, although rarely described. We highlight a case of acute pancreatitis in a female induced by levofloxacin. She presented with typical signs and symptoms of acute pancreatitis and had been taking levofloxacin for urinary tract infections for the last 3 days. After ruling out all other possible causes, her clinical picture, laboratory results, and imaging findings confirmed acute pancreatitis induced by levofloxacin.

## 1 INTRODUCTION

Pancreas is an important viscera of the endocrine system. It is vitally important in human life. However, the pancreas is vulnerable to the harmful effects of toxic agents, pathogens, and drugs. Pancreatic injury can lead to diabetes and acute pancreatitis.^1^ It is an inflammation of the pancreatic parenchyma manifested as upper abdominal pain radiating to the back, anorexia, nausea, vomiting, diarrhea, and pyrexia. It is diagnosed clinically, along with laboratory investigations such as serum amylase and serum lipase (the most specific test) and imaging modalities, including bedside abdominal ultrasonography and computed tomography (CT).^2^

The article "Acute pancreatitis associated with the antibiotic levofloxacin: A rare case report" was retracted in 2026. Reasons: plagiarism; overlap with other authors' work.

Levofloxacin belongs to a class of fluoroquinolone antibiotics used for treating intraabdominal infections, urinary tract infections, respiratory tract infections, and skin and soft tissue infections.^3^ Levofloxacin is generally well‐tolerated; however, levofloxacin is associated with photosensitivity, hypersensitivity reactions, liver toxicity, tendinitis, and tendon rupture.^4^ Levofloxacin also has a toxic effect on pancreatic tissue inducing acute pancreatitis, which is rarely described in the literature.^5^ A few cases have been published on levofloxacin as an etiology of acute pancreatitis. We report a case of levofloxacin‐induced acute pancreatitis.

## 2 CASE PRESENTATION

A 44‐year‐old female with a past medical history of hypothyroidism and diabetes mellitus presented with abdominal pain and vomiting for the last 3 days. The pain was described as an aching, crampy pain that was diffuse and located in the epigastric region and radiating to the back between the shoulder, which was not relieved by antacids or food. She also complained of nausea and multiple episodes of watery, non‐bilious projectile vomiting for the past 3 days. She described that she had been taking levofloxacin for a urinary tract infection (UTI) for the last 3 days, diagnosed on urine analysis. She had been taking amlodipine for hypertension and insulin for diabetes and was compliant with her medications. She reported no history of alcohol consumption, drug abuse, or medications other than diabetes and hypertension. She had no history of trauma or any history of pancreatitis, or similar symptoms.

On examination, she appeared uncomfortable and was clutching her abdomen. She was hemodynamically stable with blood pressure (100/70 mmHg), respiratory rate (21/min), and heart rate (99/min). Her abdomen was tender to palpate in the epigastric region with no rigidity or guarding. Bowel sounds were present, and no visceromegaly was appreciated. The rest of the systemic examination was unremarkable. Her initial laboratory evaluations revealed elevated serum lipase and amylase levels suggestive of acute pancreatitis (Table 1).

**TABLE 1:** Results of initial laboratory parameters.

Parameter	Initial lab value on admission	Lab value after drug discontinuation	Reference range
White cell count	11,000/mm^3^	10,000/mm^3^	(4000–11,000)
Hemoglobin	11 g/dL	10.2 g/dL	(13–15)
Bilirubin	0.5 mg/dL	0.5 mg/dL	(0.1–1.2)
Amylase	990 IU/L	112 IU/L	(30–110)
Lipase	1311 IU/L	170 IU/L	(0–155)
Serum creatinine	1.1 mg/dL	1.1 mg/dL	(0.7–1.3)
Serum calcium	9.9 mg/dL	9.4 mg/dL	(9.0–10)
Blood urea nitrogen	19 mg/dL	20 mg/dL	(07–26)
Alanine aminotransferase	49 IU/L	47 IU/L	(8–57)
Aspartate Aminotransferase (AST)	39 IU/L	10–40 IU/L	
Triglycerides (TG)	70 mg/dL	<150 mg/dL	
Alkaline phosphatase	77 mg/dL	70 mg/dL	(36–95)
C‐reactive protein	3 mg/dL	1 mg/dL	(0.4–1.1)
Erythrocyte sedimentation rate	31/h	20/h	(<21)

An abdominal ultrasound demonstrated a non‐distended gallbladder without wall edema and thickening; the pancreas was not visualized. Abdomen CT was performed, which showed diffuse and generalized enhancement of the pancreas with ill‐defined borders and fat stranding, and localized edema. No gallstone, biliary sludge, pseudocyst, or biliary tract abnormality was appreciated (Figure 1). Other lab evaluations were unremarkable, including a fasting lipid profile, serum triglyceride and calcium levels. Viral serology tests involving hepatitis B, C, human immunodeficiency virus, and coronavirus disease 2019 (COVID‐19) were negative to rule out an infectious cause of acute pancreatitis. Based on clinical, serological, and imaging modalities, a provisional diagnosis of acute pancreatitis induced by levofloxacin was made after ruling out all other possible causes. She met all three criteria as per the revised Atlanta classification (acute epigastric pain, elevated lipase greater than three times the normal limit, and characteristic imaging findings) for AP. Based on her CT scan findings, she met the criteria for Balthazar grade C (CT severity index: 2), which was consistent with mild AP.

The article "Acute pancreatitis associated with the antibiotic levofloxacin: A rare case report" was retracted in 2026. Reasons: plagiarism; overlap with other authors' work.

**FIGURE 1:** Abdomen computed tomography revealing pancreatic diffuse enlargement with vague borders and fat stranding.

Immediately, levofloxacin was discontinued, and she was kept oral‐free and was managed conservatively with bowel rest, intravenous fluids, appropriate analgesia, antiemetic, and proton pump inhibitor. For a urinary tract infection, she was started on fosfomycin. Over the 40 h, her symptoms started improving with the resolution of serum lipase and amylase level. She was discharged on day four with a regular follow‐up with her physician. On her follow‐up visit 2 weeks later, she was doing well.

## 3 DISCUSSION

Drug‐induced acute pancreatitis is estimated to account for 5% of all acute pancreatitis cases, and the global incidence is crossing 50–800 per one million adults.^6^ Drug‐induced acute pancreatitis can be considered the third common cause of acute pancreatitis after ruling out alcohol and gallstones.^7^ Diuretics, valproic acid, and azathioprine are commonly associated with drug‐induced acute pancreatitis. Many medications have been listed as an etiology of acute pancreatitis, including antihypertensives, antifungal, antiviral, and antibiotics.^8^ Levofloxacin as an etiology of acute pancreatitis is uncommon, and the number of cases reported is few in numbers. The incidence of levofloxacin‐induced acute pancreatitis is not yet identified as only limited data are available. Most of the cases are published as case reports. Neto et al. highlighted a case of acute pancreatitis in an old male induced by levofloxacin. He had taken levofloxacin for acute cystitis for the last 2 days.^9^ Rekhi et al.^10^ reported a case of levofloxacin‐induced acute pancreatitis in a young patient. She was commenced on levofloxacin due to pneumonitis.

The article "Acute pancreatitis associated with the antibiotic levofloxacin: A rare case report" was retracted in 2026. Reasons: plagiarism; overlap with other authors' work.

Acute pancreatitis is manifested by elevated levels of serum amylase and lipase enzymes in the body. Laboratory findings should be concomitant with the histopathological findings of pancreatic tissue. The levels of serum lipase more than two times normal are the most appropriate diagnostic marker for acute pancreatitis.^5^ However, increased levels of amylase are not diagnostic because the amylase enzyme is also secreted by the salivary glands, but the lipase enzyme is only secreted by pancreatic tissues.^11^ The mechanism of drug‐induced pancreatitis is the involvement of a toxic metabolite or a drug that either directly affects the biochemistry of the pancreatic cells or triggers an immune response against normal pancreatic tissue that further damages the structure and integrity of pancreatic tissues.^12^ Both mechanisms result in necrosis of the pancreatic cells leading to acute pancreatitis. The lipid peroxidation pathway is the most important pathway behind both these mechanisms. It is also observed that reactive oxidative stress has a major role in vancomycin‐associated nephrotoxicity. The pathophysiology includes an increased concentration of cellular adenosine triphosphate (ATP) and oxidative phosphorylation that leads to the high production of free radicals inside the cells. This production can happen either directly or indirectly.^13^

The patient presented with classic symptoms of acute pancreatitis, but due to the rarity of the cause, that is, levofloxacin as a culprit of pancreatitis, the diagnosis was delayed, although levofloxacin was stopped immediately, and the patient was appropriately managed, which alleviated the patient's condition. Physicians should rule out every possible cause to reach a definitive diagnosis.^14^

## 4 CONCLUSIONS

Levofloxacin or drug‐induced pancreatitis is a diagnosis of exclusion and is generally reached after taking a detailed patient history and performing a physical examination to rule out other important causes of pancreatitis. The diagnosis is generally delayed as this is one of the rare causes of pancreatitis. Drug‐induced pancreatitis usually damages the pancreas either through the generation of toxic metabolites or by triggering an immune response against normal pancreatic tissue. In most cases, the patient gets stable, and the pain alleviates after cessation of the offending agent and starting appropriate treatment.

The article "Acute pancreatitis associated with the antibiotic levofloxacin: A rare case report" was retracted in 2026. Reasons: plagiarism; overlap with other authors' work.

## AUTHOR CONTRIBUTIONS

**Pugazhendi Inban:** Validation. **Virali Gulla:** Conceptualization. **Aarfa Devani:** Software. **Chinaza Mercy Akuma:** Investigation. **Chengala Ananyaa Gowthavaram:** Funding acquisition. **Akbar Hussain:** Resources. **lynn lat lat aung:** Conceptualization. **Neel Jadav:** Investigation. **Bansi Savaliya:** Project administration. **Taha Sajjad:** Writing – original draft; writing – review and editing. **Aadil Mahmood Khan:** Project administration. **Ogbonnaya Akuma:** Data curation. **Anasonye Emmanuel Kelechi:** Formal analysis.

## FUNDING INFORMATION

The authors declare that they have no known competing financial interests or personal relationships that could have appeared to influence the work reported in this paper.

## CONFLICT OF INTEREST STATEMENT

The authors declare no competing interests.

## CONSENT

Written informed consent was obtained from the patient to publish this report in accordance with the journal's patient consent policy.

## Data Availability

The case report's pertinent data are available from the corresponding author upon reasonable request.
